The article "The role of expression imbalance between adipose synthesis and storage mediated by PPAR-γ/FSP27 in the formation of insulin resistance in catch up growth" was published in 2016. Journal: Lipids Health Dis.

# The role of expression imbalance between adipose synthesis and storage mediated by PPAR-γ/FSP27 in the formation of insulin resistance in catch up growth

**DOI:** 10.1186/s12944-016-0319-z

**Published:** 2016-10-04

**Authors:** Su-Xing Wang, Jin-Gang Wei, Lu-Lu Chen, Xiang Hu, Wen Kong

**Affiliations:** 1 The Second Department of Geriatrics, Hebei General Hospital, Shijiazhuang, 050051 China; 2 Department of general surgery, The fifth hospital of Shijiazhuang City, Shijiazhuang, 050024 China; 3 Department of Endocrinology, Union Hospital, Tongji Medical College, Huazhong University of Science and Technology, Wuhan, 430022 China

**Keywords:** Adipose synthesis and storage imbalance, Catch up growth, Insulin resistance

## Abstract

**Background:**

Catch up growth (CUG) motivated by under-nutrition can lead to insulin resistance (IR) and visceral fat over-accumulation. However, the precise mechanisms on IR induced by adipose tissue changes during CUG remain unresolved.

**Methods:**

Experimental rats were divided into three groups: normal chow group, catch up growth group and resveratrol administrated group. The whole experiment was carried out in four stages: 4, 6, 8 and 12 weeks.

Peroxisome-proliferator activated receptor gamma (PPAR-γ) and fat-specific protein 27 (FSP27) expression level in epididymal adipose tissues (EAT) and subcutaneous adipose tissues (SAT) were detected along with other IR indicators.

**Results:**

Calorie restriction (CR) significantly increased PPAR-γ expression in EAT while decreased FSP27 expression. During re-feeding, both of the expression of PPAR-γ and FSP27 increased, even FSP27 returned to normal level when CUG for 4 weeks. Although PPAR-γ expression declined slightly at 8 weeks, it was still much stronger than normal chow groups. However, no changes were seen in SAT. Relative insufficiency of FSP27 expression in EAT results in a decrease in lipid storage capacity, causing a series of path physiological changes that led to the formation of IR. Resveratrol inhibited the expression of PPAR-γ and promoted FSP27 expression, thus fundamentally improving IR.

**Conclusions:**

The imbalance between adipose synthesis and storage mediated by PPAR-γ / FSP27 in the EAT plays a pivotal role in the formation of IR during CUG. Resveratrol can correct fat formation and storage imbalance status by up-regulating FSP27 and down-regulating PPAR-γ expression level, ameliorating insulin sensitivity.

## Background

Nutritional rehabilitation after malnutrition could motivate catch up growth, which has been characterized by rapid growth after a temporary period of growth retardation and apparent insulin resistance and an accelerated rate of fat storage [1, 2]. Redistribution of glucose from skeletal muscle to adipose tissue [3] and increased adipose tissue lipid synthesis ability [4] enhance conversion of glucose to lipids in fat stores, eventually leading to fat catch up preferentially [4]. Adipose tissue is recognized as key contributor to the systemic insulin resistance and overt diabetes seen in metabolic syndrome [5]. However, lipid synthesis enhancement alone does not necessarily cause IR, as evidenced by good insulin sensitivity in a few obese persons [6]. Moreover, the thiazolidinediones which are selective ligands for the nuclear transcription factor peroxisome proliferator-activated receptor (PPAR) γ [7] can improve IR partially by promoting the storage of triacylglycerol in adipocytes, thus decreasing ectopic lipid deposition and enhancing insulin sensitivity [8]. Therefore, the formation of IR during CUG is not completely explained merely by an improvement in lipogenesis and increased fat content. Other pathways by which changes in adipose tissue occur should be explored.

Recent research has demonstrated that fat storage capacity might represent a contributing factor in the varying degrees of insulin resistance observed among obese human subjects, with an inverse correlation between fat storage capacity and insulin resistance [6]. Efficient storage of excess fatty acids within adipocyte lipid droplets serves to protect other cells and tissues from their lipotoxic effects [9, 10] reducing the risk of IR occurrence. Adipocytes express high levels of two distinct lipid droplet proteins, FSP27 (also called CIDEC), a member of the CIDE family, and perilipin1 (PLIN1), a member of the PAT family [11, 12]. The C-terminus domain, aa 120–220, of FSP27 interacts with PLIN1 to regulate lipid droplet size in adipocytes [12], and PLIN1 acts as a scaffold for FSP27 at the LD surface where FSP27 facilitates the fusion of LDs [13]. Compared to PLIN1, studies have confirmed that caloric restriction reduced the expression of FSP27 [14], according to the experimental design and intention, we explored changes in FSP27 during CUG.

As shown previously, lipogenesis key gene PPAR-γ is markedly enhanced in the CUG process [4]. PPAR-γ, which is a master regulator of adipogenesis [15, 16], belongs to the nuclear receptor super-family of ligand-activated transcription factors and plays a pivotal part in lipid biosynthesis [16]. Genes regulated by PPAR-γ are diferentially regulated not only by agonist binding but also by phosphorylation of the ligand binding domain of PPAR, including Acyl, aP2, Plin1, C/EBPα and other genes, up to dozens of species [17–20]. It has been suggested that loss of PPAR-γ expression in murine embryonic fibroblasts leads to a complete absence of adipogenic capacity [21]. As is known to all, nutrition deficiency is the main driving factor of CUG, previous studies have suggested that CR can increase adipose tissue expression of PPAR-γ [22, 23], and also affects fat storage capacity. Magnusson et al. found that CR could significantly reduce the FSP27expression [14]. We therefore postulate that the opposite changes in PPAR-γ and FSP27 during CUG motivated by CR may be the main reason of the formation of IR.

Resveratrol, a polyphenol found in red wine that is associated with a surprising number of health benefits [24], can ameliorate IR [25, 26]. Previous studies have demonstrated that PPAR-γ is closely associated with IR [27]. Resveratrol negatively modulates PPAR-γ protein levels [28] through activating SIRT-1 deacetylase activity [29, 30]. However, to our knowledge, no previous studies have addressed how resveratrol influences FSP27 in adipose tissue. Therefore, in this study, we investigated whether resveratrol can effectively correct the PPAR-γ/FSP27 ratio in CUG rats.

Briefly, the general objectives of this study were three fold. The first was to explore the mechanism of IR induced by adipose tissue, including changes in PPAR-γ/FSP27 ratio and relevant indicators of IR during CUG process. The second aim was to compare the effects of resveratrol intervention on PPAR-γ/FSP27. Finally, we assessed the role of expression imbalance between adipose synthesis and storage mediated by PPAR-γ/FSP27 in the formation of IR in CUG model.

## Methods

### Animals and diets

Fifty-four healthy male Sprague–Dawley rats weighing 140–180 g were purchased at 6 weeks of age, (Center of Experimental Animals, Tongji Medical College, Huazhong University of Science and Technology, China, SCXK (E) 2010–0009) and acclimatized for 1 week. The animals were individually housed in stainless steel cages with free access to standard chow pellets and water, under uniform housing in environmentally controlled conditions (22 ± 2 °C, 12-h light–dark cycle, and 55–65 % humidity). The calorie of normal chow contained 14 % fat, 64 % carbohydrate, and 22 % protein (per 100 g: 6.9 g fat, 69.3 g carbohydrate, 23.8 g protein), which was provided by the Laboratory Animal Center of Tongji Medical College mentioned above. All protocols of animal treatment were approved by the institutional animal ethics committee.

### Experimental design

The rats were randomly divided into three groups: normal chow group (NC group, containing NC4, NC8 and NC12 subgroups); catch up growth group (CUG group, containing three subgroups RN2, RN4 and RN8); catch up growth with resveratrol administrated group (CUGE group, containing R4E and RN8E subgroups). The whole experiment was carried out in four stages: 4, 6, 8 and 12 weeks, and statistical analysis was conducted on the related indexes of the experimental animals with the same growth period (NC4, R4 and R4E; NC8 and RN4; NC12, RN8 and RN8E) (Table 1). The animals in the CUG and CUGE groups were restricted to 60 % of the normal chow consumption of their counterparts in the control groups for four weeks (R4) and then were re-fed for 2, 4 or 8 weeks. During this time, food intake was strictly matched with that of pair-fed controls, to avoid the hyperphagic response (RN versus NC). To study adipose synthesis and storage changes in the whole experimental process, we detected related parameters at the end of the caloric restriction (R4) groups. Resveratrol (Sigma, St Louis, MO) mixed with saline solution (0.9 % normal saline, NS) was administered orally by gavage in R4E (4-week CR plus resveratrol intervention) and RN8E groups (the same dietary pattern as with RN8 plus resveratrol treatment, that is, resveratrol intervention after 4-week CR) (100 mg/kg/d). The other groups received a corresponding volume of saline solution every day. Taken together, this study contained nine subgroups, and each subgroup contained six animals (Table 1).

**Table 1:** Primer design for genes analyzed by real-time PCR

SYBR Green RT-PCR Primers	Forward Primer	Reverse primer	Annealing temperature
PPAR-γ	TGTCGGTTTCAGAAGTGCCTTG	TTCAGCTGGTCGATATCACTGGAG	60 °C
FSP-27	AAGGCATCATGGCCCACAG	TCTCCACGATTGTGCCATCTTC	58 °C
SIRT-1	TCCTCACTAATGGCTTTCATTCCTG	GTGCCAATCATGAGATGTTGCTG	57 °C
β-Actin	GGAGATTACTGCCCTGGCTCCTA	GACTCATCGTACTCCTGCTTGCTG	62 °C

### Body weight and body fat measurement by DEXA

Body weight in experimental 4 and 12 weeks subgroups (including NC4,

R4, R4E, NC12, RN8, RN8E groups) was measured every day. Whole-body composition was measured by dual-energy X-ray absorptiometry (DEXA) with a scanner (Lunar prodigy advanced, GE Company) by the same experienced technician. At the end of 4 and 12 experimental weeks (Fig. 1), rats were first anesthetized by intraperitoneal injection of pentobarbital (30 mg/kg body weight) and were then were placed in supine position, both upper and lower extremities extended, and fixed to the examining table (Fig. 2, which was collected in the automatic imaging of the machine). Fat content of torso tissue and whole body tissue, and the ratio of torso fat to whole body fat were determined.

**Fig. 1:** The experimental design, each subgroup included 6 rats

**Fig. 2:** Photograph of body fat measurement by DEXA

### Hyperinsulinemic–euglycemic clamp in conscious status and measurement of in vivo 2-deoxy-D-glucose (2-DG) uptake in adipose tissue

A 120-min hyperinsulinemic–euglycemic clamp in conscious rats based on tail artery measurement of 2-DG (Sigma-Aldrich, St Louis, MO) uptake in adipose tissue was determined as described previously [1]. Blood samples (20 μl) were collected every five minutes for plasma glucose determination using a glucometer (One Touch Ultra, Lifescan, Milpitas, CA, USA). The average glucose infusion rate between the 60th and 120th minute (GIR_60–120_) was used to evaluate systemic insulin sensitivity.

### Hematoxylin and eosin (H & E) staining

Fresh tissues (epididymal adipose tissues) were collected and fixed in 4%neutral buffered formalin solution (HT50-1-2; Sigma). The tissues were then embedded in paraffin, cut into 4 *μ*m thick sections, mounted on glass slides, and stained with hematoxylin and eosin solution (H & E), and processed according to standard procedure.

### Adipose tissue SIRT1 Activity determination

Enzyme activity assay of SIRT1 was carried out using a commercial kit (Genmed Scientifics) as described before [25].

### RNA extraction and real-time RT-PCR

Total RNA was extracted from the epididymal and subcutaneous adipose tissue using Trizol reagent (RNAiso™ Plus, TaKaRa Code D9108B, Japan) according to the manufacturer’s protocol. The quantity and quality of the total RNA was verified with a spectrophotometer. The process of synthesizing single-stranded complementary DNA and target gene amplification was carried out as previously reported [25]. Real time PCR reactions were conducted in an ABI 7900 HT apparatus (Applied Biosystems) in triplicate. Specific kits used were as follows: 2-step RT-PCR: Prime Script ® RT Master Mix Perfect Real Time, TaKaRa Code DRR036S, Japan; Real-Time PCR System: SYBR Green I dye (TaKaRa Code DRR420A, Japan). Relative expression levels were calculated using the comparative Ct (2^−ΔΔCt^) method with β-actin RNA as the endogenous control. Oligonucleotide sequences of forward and reverse primers are shown in Table 1.

### Western blot analysis

Western blot analysis was performed to determine target protein expression including adipose formation and storage proteins (PPAR-γ, FSP27). Total proteins were extracted from adipose tissue samples using a Total Protein Extraction kit (Beyotime, Shanghai, China) according to the manufacturer’s instructions. Took adipose tissue samples, weighed, according to the proportion of weight: volume = 1:6 to add protein lysis solution, full grinding. Total protein concentration was calculated by BCA protein reagent (Pierce, Rockford, IL, USA), and the concentration was not less than 2 μg/μl. Then, 60 μg of protein lysate per sample was determined. Proteins were then separated by sodium dodecyl sulfate polyacryl-amide gel electrophoresis and transferred to PVDF membrane.

The membrane was incubated with appropriate polyclonal primary antibodies (Cell Signaling Technology, USA) (PPAR-γ and FSP27 antibody, 1:3000 and 1: 1500 diluted in 5 % non-fat milk, respectively). All Western blots shown were representative of at least two independent experiments and quantified by densitometry analysis.

### Blood sample detection

Plasma adiponectin, TNF-α concentrations and basal insulin were measured with enzyme-linked immunosorbent assays with commercial kits (Westang Biotechnology, Shanghai, China; Linco RIA rat insulin kit, St Charles, MO). Serum free fatty acid (FFA) and triglyceride (TG) levels were performed by a colorimetric enzymatic method (Wako nonesterified fatty acid C kit, Richmond, VA, and GPO-PAP, Roche Diagnostics, Indianapolis, IN).

### Statistical analysis

All analyses were performed with the Statistical Package for Social Sciences version 16.0 (SPSS, Chicago, IL). Results were presented as the mean ± SD. Differences in bone parameters among groups were investigated using one-way analysis of variance (ANOVA). Statistical significance level was considered at *P* < 0.05.

## Results

### Body weight and body fat distribution

During the four-week diet restriction period, body weight of rats decreased significantly compared with the NC4 group. After re-feeding for 8 weeks, it was still consistently lower than the normal level (*P* < 0.05, RN8 vs. NC12) (Fig. 3a). Food restriction induced a slight increase in fat content of torso tissue and whole body tissue, and in the ratio of torso fat/whole body fat in R4 group, but the values did not reach statistical significance compared to NC4 group (Fig. 3b-d). Following the 8-week catch up growth, fat content of torso and whole body tissue significantly increased, meanwhile torso fat/ whole body fat ratio also distinctly increased compared with NC12 group (*P* < 0.01) (Fig. 3b-d). However, in resveratrol intervention groups, body weight and body fat content was significantly lower than the control groups (R4E vs. R4, RN8E vs. RN8), and body fat content in the RN8E group was virtually reduced to or far below normal level in the R4E group (Fig. 3a-d).

**Fig. 3:** Comparisons of body weight (**a**) and fat content (**b**, **c**, **d**) Pre- and Post- resveratrol treatment. Food restriction induced a significant decrease in body weight, after re-feeding for 8 weeks, it was still consistently lower than the normal level, but fat content of torso and whole body tissue significantly increased. After resveratrol intervention, body weight and body fat content was significantly lower than the control groups. † *P* < 0.05 versus NC_4_ group, § *P* < 0.01 versus NC_4_ group. △*P* < 0.05 versus R4 group, ▲*P* < 0.01 versus R_4_ group. *P < 0.05 versus NC_12_ group, #*P* < 0.01 versus NC_12_ group. ☆*P* < 0.05 versus RN_8_ group, ★*P* < 0.01 versus RN_8_ group

### Systemic and adipose tissue insulin sensitivity

Fasting blood glucose (FBG) and fasting insulin (FINS) levels did not change significantly in R4 groups (*P* > 0.05, R4 vs. NC4). CUG led to a non-significant increase in FBG levels (*P* > 0.05, RN8 vs. NC12). FINS levels were notably increased in RN8 group (*P* < 0.01, RN8 vs. NC12) (Fig. 4a, b). Food restriction induced a slight increase in the average GIR_60–120_ at hyperinsulinemic-euglycemic clamp, but it was not statistically significant compared with the normal group. However, the average GIR_60–120_ decreased significantly in the RN8 group (*P* < 0.05, RN8 vs. NC12) (Fig. 4c). Distinctly increased FINS levels and decreased GIR_60–120_ induced by CUG indicated systemic IR. In addition, insulin-stimulated glucose uptake in epididymal adipose tissue was increased by diet restriction (∼15 %, R4 vs. NC4, *P* <0.01), and this increase was further enhanced in CUG (∼29 %, *P* < 0.01, RN8 vs. NC12) (Fig. 4d). However, although glucose uptake in subcutaneous tissue was also increased during diet restriction and CUG, the changes were less remarkable compared to those seen in epididymal adipose tissue (Fig. 4e). Resveratrol treatment decreased FINS levels, and increased GIR_60–120_ and adipose tissues glucose uptake as shown in CUG group (*P* <0.01, RN8E vs. RN8) (Fig. 4b-e). However, only adipose tissue glucose uptake was increased in R4E group. FINS levels and GIR_60–120_ were not altered (Fig. 4a-e). We also found that resveratrol had little effect on FBG (Fig. 4a).

**Fig. 4:** FBG (**a**), FINS (**b**), GIR_60–120_ levels (**c**), and 2-DG uptake (**d**, **e**) Pre- and Post- resveratrol treatment. Hyperinsulinemic-euglycemic clamp showed that fasting blood glucose, fasting insulin and GIR_60–120_levels did not change significantly in R4 groups, CUG led to a significant increase in FINS levels and decrease GIR_60–120_ in epididymal adipose tissue. Resveratrol treatment decreased FINS levels, increased GIR_60–120_ and adipose tissues glucose uptake as shown in CUG group. §*P* < 0.01 versus NC_4_ group, △*P* < 0.05 versus R_4_ group. ▲*P* < 0.01 versus R_4_ group, *P < 0.05 versus NC_12_ group. #*P* < 0.01 versus NC_12_ group, ☆*P* < 0.05 versus RN_8_ group. ★*P* < 0.01 versus RN_8_ group

### The morphology of epididymal adipocyte

In investigating the cell size of the epididymal adipose, we found that the diameter of adipose cells in the R4 group was smaller than in the control group (*P* < 0.01, R4 vs. NC4) (Fig. 5a, b); while in the RN8 group adipose cell’ diameter was obviously larger, with abnormal shape, appearing fused with each other (*P* < 0.01, RN8 vs. NC12) (Fig. 5d, e). Resveratrol decreased the size of adipocytes observed in R4E and RN8E groups and protected the integrity of cell membranes (*P* <0.01, RN8E vs. RN8, R4E vs. R4) (Fig. 5c, f).

**Fig. 5:** HE staining of epididymal adipocytes in each group (400×). Food restriction made epididymal adipocytes significantly smaller, after CUG adipose cell’ diameter was obviously larger, with abnormal shape. Resveratrol decreased the size of adipocytes and protected the integrity of cell membranes. §*P* < 0.01 versus NC_4_ group, ▲*P* < 0.01 versus R_4_ group. ★*P* < 0.01 versus RN_8_ group

### Alteration of SIRT1 activity and mRNA analysis in adipose tissue

The R4 rats showed more than a 30 % increase (*P* < 0.01) in epididymal and subcutaneous adipose SIRT1 activity, but a significant reduction was observed in the RN8 group compared with the control rats (31 % ∼ 35 %, *P* < 0.01) (Fig. 6a, b). Conversely, oral administration of resveratrol distinctly improved SIRT1 activity, which either matched or exceeded NC group when the 8-week re-feeding ended (Fig. 6a, b). SIRT1 real-time RT-PCR analysis was consistent with the activity results real-time RT-PCR analysis was consistent with the activity results (Fig. 7e).

**Fig. 6:** Alteration SIRT1 activity in epididymal (**a**) and subcutaneous (**b**) adipose tissue. The R4 rats showed a significant increase in SIRT1 activity in adipose tissue, but an obvious reduction in the RN8 group. Oral administration of resveratrol distinctly improved SIRT1 activity. §*P* < 0.01 versus NC4 group, ▲*P* < 0.01 versus R4 group. #*P* < 0.01 versus NC12 group,☆*P* < 0.05 versus RN8 group,★*P* < 0.01 versus RN8 group

**Fig. 7:** Comparisons of the expression data (2Ct-values) in adipose tissue. The expression of PPAR-γ mRNA did not change significantly in subcutaneous adipose (**b**), food restriction made PPAR and FSP27 mRNA expression change in different side, after catch up growth the two mRNA expression were significantly higher than normal group. Resveratrol obviously inhibited PPAR mRNA expression, but increased FSP27 expression (**a**, **c**, and **d**); SIRT1 mRNA expression in epididymal adipose tissue was consistent with the activity results (E). §*P* < 0.01 versus NC_4_ group, ▲*P* < 0.01 versus R_4_ group, #*P* < 0.01 versus NC_12_group, ★*P* < 0.01 versus RN_8_ group, △*P* < 0.05 versus R_4_ group

### Inconsistent expression levels of PPAR-γ and FSP27 in CUG

To investigate the changes of adipose formation and storage capacity during CUG, we analyzed PPAR-γ and FSP27 mRNA and protein expression levels. Western blot analysis of epididymal adipose tissue suggest that diet restriction increased PPAR-γ expression but suppressed FSP27 expression compared with normal group (Fig. 8a). After re-feeding, PPAR-γ expression levels increased significantly, and achieved the highest level at CUG of 4 weeks. Although it decreased to some degree at the end of the experiment, it was still far higher than the NC_12_ group (Fig. 8a). These results were consistent with FSP27 and PPAR-γ mRNA expression (Fig. 7a). Relative to PPAR-γ, low level protein expression of FSP27 induced by diet restriction gradually increased and virtually recovered to normal levels after re-feeding for 4 weeks, then exceeded the NC group when the experiment ended (Fig. 8a). However, the alteration of PPAR-γ expression levels was not obvious during the CUG process in subcutaneous adipose tissue (Figs. 7b and 8b), and, thus, we did not detect FSP27 expression levels in this tissue. Both PCR and western blot analysis indicated that resveratrol treatment markedly reduced epididymal adipose tissue PPAR-γ expression (Figs. 7c and 8c), but up-regulated FSP27 expression levels (Figs. 7d and 8d). SIRT1 expression levels also were up-regulated in epididymal adipose tissue (Fig. 7e).

**Fig. 8:** Comparisons of the PPAR-γ and FSP27 protein expression Pre-(**a**, **b**) and Post-(**c**, **d**) resveratrol intervention. PPAR-γ and FSP27 protein expression levels and the effect of resveratrol intervention in epididymal adipose tissue were consistent with mRNA changes (Fig. 7a, c, d). *P < 0.05 versus NC12 group, #*P* < 0.01 versus NC_12_group, †*P* < 0.05 versus RN_8_ group, ▲*P* < 0.01 versus RN8 group. △*P* < 0.01 versus R_4_ group

### Serum FFA /TG and Plasma TNF-α/ adiponectin concentrations

Compared with the control, blood lipid FFA (Fig. 9c) was increased and TG (Fig. 9d) was lower in the diet restriction stage, but both of them were significantly elevated in RN8 group. The levels of TNF-α did not change significantly during the diet restriction period compared to NC group, while they were markedly increased in the RN8 group (Fig. 9a). However, adiponectin levels, which changed inversely with TNF-α, increased because of diet restriction but decreased significantly during CUG (Fig. 9b). Resveratrol treatment had no major impact on blood lipid levels (Fig. 9c, d), but decreased TNF-α levels and increased adiponectin levels in the experimental rats (Fig. 9a, b).

**Fig. 9:** Comparisons of blood sample during CUG and with resveratrol intervention. Adiponectin and TNF-α levels changed inversely during CUG (**a**, **b**), FFA and TG levels were significantly elevated in RN8 group (**c**, **d**). Resveratrol treatment had no major impact on blood lipid levels (**c**, **d**), but decreased TNF-α levels and increased adiponectin levels (**a**, **b**). † *P* < 0.05 versus NC_4_ group, §*P* < 0.01 versus NC_4_ group. △*P* < 0.05 versus R_4_ group, #*P* < 0.01 versus NC_12_group. ☆*P* < 0.05 versus RN_8_ group, ★*P* < 0.01 versus RN_8_ group

## Discussion

Adipose tissue is an important metabolic organ that is crucial for whole-body insulin sensitivity and energy homeostasis, and IR states. Compared to other parts adipose tissue of the body, visceral adipose tissue plays an important role in IR [31]. Lipids synthesis and storage are affected by many factors, among them, the nuclear hormone receptor PPAR-γ is a central regulator of adipogenesis and plays a dominant role in fat tissue development [15, 16]. FSP27/Cidec is most highly expressed in white and brown adipose tissues and increases in abundance by over 50-fold during adipogenesis [32]. Depletion of FSP27 by siRNA in murine -cultured white adipocytes resulted in the formation of numerous small lipid droplets and the almost total disappearance of large lipid droplets [33]. PPAR-γ and FSP27 play an important role in lipid synthesis and storage, so we think they can be used to assess the ability of lipid synthesis and storage to a certain extent.

In our study, 4-week diet restriction made the body weight of rats decrease significantly compared with the NC4 group. And, calorie restriction obviously increased PPAR-γ expression but suppressed FSP27 expression in epididymal adipose tissues compared with the normal group. It could be suggested that weight loss caused cellular stress in adipocytes and improved adipogenesis [34], while PPAR-γ was a central regulator of adipogenesis [15, 16], so we speculate that the weight loss caused by diet restriction stimulates lipid synthesis, and then increases PPAR-γ expression. Similarly, other studies also observed that calorie restriction significantly increased the expression of PPAR-γ [22, 23]. There is less research on the relationship between calorie restriction and FSP27. Our data indicated that calorie restriction obviously suppressed FSP27 expression in epididymal adipose tissues. Similar observations had been made by Magnusson [14]. We speculate that it is the decrease in caloric intake per se that leads to reduced FSP27 expression. Whether there are other genes involved in the regulation is not clear, and needs further study. In addition, the expression of PPAR-γ and FSP27 did not return to normal level after 8-week catch up growth, which was possibly related to the short observation time. This study showed that calorie restriction led the expression of PPAR-γ and FSP27 to appearing the opposite trend. However, recent studies demonstrate that FSP27 gene is a direct downstream target of PPAR-γ and specifically regulated by PPAR-γ [35]. This seemingly contradictory change between the two genes caused by calorie restriction can be explained by the fact that nutrition substrate may play a major role during this process, because the expression of many adipocyte-specific genes is affected by dietary manipulations [36]. Due to inadequate nutrient substrate supply, down-regulation of FSP27 might be part of an adaptation by the adipocyte to whole-body energy deficiency [23], resulting in reduced lipid storage. In our study, although the capability of adipogenesis mediated by PPAR-γ increased due to calorie restriction, it only showed a potential and could not be exerted because of energy deficiency. Once the supply of nutrients was adequate as was the case during re-feeding, both PPAR-γ and FSP27 showed the same tendency, and increased to different degrees. Although fat storage capability (FSP27) was gradually enhanced and even exceeded NC at the end of the experiment, it was still relatively deficient compared to the continued up-regulation of fat synthesis capability (PPAR-γ). Based on the above observations, we reason that the inconsistent changes of lipid generation and storage caused by under-nutrition are the primary reason for IR formation during CUG.

Similar to the previous studies [1, 3], our CUG models showed the accelerated rate of fat recovery. Although body weight in RN8 group was still lower than the normal levels, DEXA results indicated that fat content of torso and torso fat/ whole body fat ratio in RN8 distinctly improved compared with NC group. We speculated that insulin-stimulated increase of glucose uptake in adipose tissue of RN8 group enhanced the availability of raw materials for fat synthesis. Additionally, FSP27 expression increased compared to NC at the end of re-feeding for 8 weeks despite it still being relatively lower than PPAR-γ, and the improved lipid storage capacity promoted the fat accumulation. Eventually, all of these changes led to the catch up of fat. Nevertheless, it is to be noted that food-restricted rats had a slight increase in fat content of torso tissue and whole body tissue in this study. We speculated that brief calorie restriction (4 weeks) increased PPAR-γ expression, while PPAR-γ could promote the uptake of FFAs and increased the content of TAGs in the adipocytes [37], and thereby improved the body fat content [37]. Epidemiological as well as other evidence indicate that abdominal fat is more directly related to negative health outcomes than that of subcutaneous fat [38]. In this study, we also noted that although CR enhanced PPAR-γ expression of SAT, the following CUG had little effect on it, which did not warrant further detection of FSP27 expression. In addition, the glucose uptake of SAT did not change significantly during CUG process compared with NC group. Therefore, our study showed that CUG had little effect on lipid synthesis of SAT, which further proved that the changes of EAT during CUG played an important role in the formation of IR. Regardless, this study is the first to observe PPAR-γ expression and glucose uptake of SAT in CUG rats. As noted above, this study reveals new insights on CUG and IR, demonstrating that the imbalance of adipose synthesis and storage mediated by PPAR-γ/FSP27 in EAT play a pivotal role.

It is well known that the hyperinsulinemic-euglycemic clamp is the criterion standard method with a high degree of accuracy to assess insulin sensitivity. In this study, the evidence of decreased steady-state GIR during the clamp in the RN8 group and significantly increased fasting insulin levels with normal fasting glucose concentration confirmed the presence of systemic IR. In addition, we found that serum FFA and TG levels were markedly elevated in the RN8 group compared with the NC group. Elevated levels of lipids such as FFAs and triglycerides are a key reason for the incidence of IR [39]. Adipocytokines are cytokines secreted by visceral adipocytes, and they are associated with metabolic syndrome and IR [40]. In our study, the levels of TNF-α increased significantly in the RN8 group compared with the NC group, However, adiponectin changed inversely with TNF-α. TNF-α is a major mediator of chronic inflammation and insulin resistance [41], and neutralization of TNF–α significantly improves insulin sensitivity [42]. Adiponectin has been related to enhanced insulin sensitivity and anti-inflammatory effect with its plasma levels negatively correlated with visceral adiposity [43]. In this study, the relative deficiency of fat storage capability could not fully store the excessive lipid that was synthesized, resulting in lipid spillover and abnormal adipokine secretion, which led to the formation of IR.

Resveratrol is a natural polyphenol produced by plants in response to environmental stress [44]. The data presented here indicated that resveratrol administration markedly restrained PPAR-γ expression and up-regulated FSP27 expression levels in EAT. The inhibitory role of resveratrol on PPAR-γ may be due to SIRT1 activation, since resveratrol is a classic SIRT-1 activator [29, 30], and SIRT1 can repress PPAR-γ in white adipose tissue by docking with its cofactor nuclear receptor co-repressor (NCoR) [30]. In our study, we observed that SIRT1 activity and mRNA expression were significantly reduced in RN8 group but distinctly improved after resveratrol administration. These results are also consistent with the changes observed with PPAR-γ. Nevertheless, the effect of resveratrol on the expression of FSP27 has not been previously reported, and only one study showed that resveratrol did not modify perilipin expression, which is another common lipid droplet-associated protein [45]. Sawada et al. found that, a competition existed in vitro between FSP27 and perilipin expression because both proteins preferentially locate to lipid droplets [46]. Therefore, we speculate that because of resveratrol up-regulation of FSP27 expression, perilipin expression promotion was not favored, which led to the observed result. The enhanced storage of triglyceride in lipid droplets of adipose tissues decreases the fatty acid levels in the circulation, thereby protecting muscle and liver from high fatty acid levels, which improves insulin sensitivity.

As noted above, adipose synthesis was in parallel with storage during CUG with resveratrol intervention, and systemic IR was improved as shown by decreased FINS levels and increased steady-state GIR in RN8E group. Although numerous studies on diabetic rats revealed the anti-hyperglycemic action of resveratrol [25], this effect was not obvious in our study. We observed that in resveratrol groups FBG was still comparable to those of the non-treatment groups in addition to a slight decrease. It was remarkable that body fat content and blood lipids (serum FFA and TG) in RN8E group were significantly decreased. Possible explanations include inhibited PPAR-γ inhibition by resveratrol through SIRT1activation [24], and increased lipolysis and reduced lipogenesis in mature adipocytes [47]. We further demonstrated that because of the relative balance of fat synthesis and storage by resveratrol treatment, plasma adiponectin was markedly increased and inflammation factor TNF-α decreased.

Mature adipocytes store triglycerides in a single fat droplet that almost entirely fills the cell [48]. Therefore, we thought the size of adipocytes would reflect the unilocular lipid droplet-size. Therefore, we studied the cell size. Results showed that adipocyte diameter in EAT was smaller during CR compared with the NC group. These small adipocytes had a high potential to store lipids, and could have improved insulin sensitivity [49]. However, during CUG, adipocytes enlarge and their shape become irregular, with incomplete cell membranes. These changes led to cell membrane rupture, lipid overflow, and serum FFA increase, and, eventually, IR. Resveratrol activated SIRT1 which then repressed PPAR-γ transactivation and inhibited lipid synthesis in adipocytes [30], at the same time enhancing lipid storage capacity. These cells had a high potential to store lipids, and, therefore, alleviate peripheral lipotoxicity. Finally, the balance between lipid synthesis and storage was restored so that fat cells were able to store excess lipid, with adipocytes’ shape and membrane almost returning to normal.

## Conclusion

In conclusion, this study has shown that CR has opposing effects on PPAR-γ and FSP27 of EAT, which becomes the main reason for the imbalance between adipose tissue synthesis and storage capacity. However, during the CUG process that followed, both of them were enhanced to varying degrees. The excessive lipid could not be stored properly, resulting in lipid spillover and causing IR. The imbalance between adipose synthesis and storage mediated by PPAR-γ/FSP27 may serve as a new molecular target for the treatment of IR and related diseases. Similar to CR, resveratrol induced upregulation of FSP27 and downregulation of PPAR-γ leading to the restoration of the balance between lipid production and storage. This provides a potential treatment for IR.

## Abbreviations

2-DG: 2-deoxy-D-glucose
CR: Caloric restriction
CUG: Catch up growth
DEXA: X-ray absorptiometry
EAT: Epididymal adipose tissues
FBG: Fasting blood glucose
FFA: Free fatty acid
FINS: Fasting insulin
FSP27: Fat specific protein 27
GIR60-120: The average glucose infusion rate between the 60th and 120th minute
H & E: Hematoxylin and eosin
IR: Insulin resistance
PPAR γ: Peroxisome-proliferator activated receptor gamma
SAT: Subcutaneous adipose tissues
TG: Triglyceride
